The article "Therapeutic Mechanism and Clinical Observation of Traditional Chinese Medicine Combined with Interventional Recanalization for Tubal Infertility" was published in 2021. Journal: Evid Based Complement Alternat Med.

# Therapeutic Mechanism and Clinical Observation of Traditional Chinese Medicine Combined with Interventional Recanalization for Tubal Infertility

**DOI:** 10.1155/2021/2842250

**Published:** 2021-10-31

**Authors:** Can Liu, Hao Qiu, Rong Huang, Hua Chai, Guibin Yuan, Shihang Shan

**Affiliations:** Department of Radiology and Imaging, The Third People's Hospital of Yunnan Province, No. 292, Beijing Road, Kunming, Yunnan 650011, China

## Abstract

To observe the clinical effect of traditional Chinese medicine (TCM) combined with interventional recanalization therapy in the treatment of tubal obstructive infertility, first, different treatment approaches were used on rabbits, and transmission electron microscopy (TEM) indicated that interventional recanalization combined with TCM can significantly ameliorate the pathological condition of the fallopian tube after treatment. Moreover, ELISA disclosed that the treatment could significantly reduce the levels of interleukin-1*β* (IL-1*β*), interleukin-6 (IL-6), and tumor necrosis factor-*α* (TNF-*α*) and increase the expression of interleukin-10 (IL-10), which demonstrated that TCM therapy can help against inflammation of the fallopian tubes. PCR array analysis revealed that BMP4, BMPR1A, SMAD2, SMAD3, SMAD4, and KLF10 expressions were upregulated, and SMAD7 expression was downregulated, proving that combined treatment could influence gene expression in the TGF-*β* family and further regulate the secretion of proteins in SMADs. In addition, a clinical study recorded the fallopian tube patency rate of 165 patients after 12 months. The recanalization rates in the two groups were 81.9% and 53.1%, with the higher rates in the combined medicine enema group. All these findings implied that interventional recanalization combined with TCM preparation has a stronger effect. The mechanism probably involves effects on the expression of genes in the TGF-*β*/SMAD and BMP/SMAD signaling pathways, with simultaneous regulation of inflammatory factors, thereby improving the ovarian environment and increasing pregnancy rates.

## 1. Introduction

In China, one out of six couples who is in reproductive age is infertile, and this number in increasing year by year [1]. Tubal infertility, the main cause of female infertility, accounts for 15.5% of cases [2, 3]. Fallopian tubal obstruction is an important cause, accounting for 25 to ∼35% of cases, and it mainly presents as infertility, along with abdominal pain and sexual pain [4]. Tubal obstruction is mostly caused by pelvic inflammatory disease (PID), including endometritis, pelvic peritonitis, and salpingitis, among which salpingitis is the most common. Inflammation is not only the main cause of tubal obstruction, but also one of the main clinical manifestations. Tubal obstruction is often accompanied by inflammation and changes in inflammatory cytokines, which are also regarded as important reference index for the diagnosis of tubal obstruction infertility [5–10].

As the most frequent gynecological disease, fallopian tubal obstruction has affected many families. Fallopian tube interventional recanalization, a new treatment method that plays a dual role in diagnosis and treatment, is minimally invasive, has low cost, and is easily accepted by patients, but the postoperative fallopian tube reocclusion rate is high. There is evidence that the recanalization rate of the procedure is approximately 90%, with a high postoperative reocclusion rate of 20–50%. Thus, traditional Chinese medicine is used as an adjuvant therapy for fallopian tube recanalization, not only shortening the treatment time, but also preventing reobstruction and improving the pregnancy rate [4, 11, 12]. Ried suggests that, compared with Western medical fertility drug therapy, management of female infertility with Chinese herbal medicine can improve pregnancy rates 2-fold within a 3–6-month period [13], and many studies have also proved it. It was pointed out that all these medicines can inhibit inflammatory exudation and accelerate the regression of inflammation, so as to promote the repair of oviduct mucosa and the regeneration of cilia, promoting blood circulation and removing blood [4, 14–16]. Although all these medicines have good curative effects, their mechanisms in the treatment of fallopian tubal obstruction are still unclear.

TGF-*β* superfamily members are a class of growth factors with a variety of biological activities, which play an important regulatory role in inflammation, tissue repair and embryonic development, cell growth, differentiation, and immune function. In recent years, TGF-*β* is widely considered to be related to chronic tubal obstructive infertility, and a large number of experiments have proved that it may be the cause of tubal adhesion. Moreover, TGF-*β*1 is an isoform of TGF-*β*, playing a key role in the development inflammation, and the expression of TGF-*β*1 in tubal intima of infertile patients with tubal obstruction was higher than that of normal population, which confirmed that it may be related to the incidence of tubal obstructive infertility [17–19].

Therefore, to develop a new treatment approach, we utilized a primary interventional therapy combined with a Chinese herbal preparation as a supplemental therapy for fallopian tubal obstruction. Different administration pathways were used in animals to investigate the mechanism of this condition. At the same time, clinical data were also assembled to provide a more detailed view.

## 2. Materials and Methods

### 2.1. Preparation of a TCM Decoction

Based on the clinical experience, we integrated the doctors' clinical experience and selected these traditional Chinese medicines. First, the TCM decoction was prepared, and the components were as follows: 30 g of each of *Angelica* sinensis (Oliv.) Diels (Danggui), *Cinnamomum cassia* Pres. (Guizhi), *Taraxacum mongolicum* Hand. -Mazz. (Pugongying), *Corydalis bungeana* Turcz. (Diding), *Sparganium stoloniferum* Buch. -Ham. (Sanleng), *Scutellaria barbata* D. Don (Banzhilian), *Curcumap haeocaulis* VaL. (Ezhu), and *Foeniculum vulgare* Mill. (Xiaohuixiang) and 15 g of each of *Hedyotis diffusa* Willd (Baihuasheshecao) and *Lonicera macranthoides* Hand.-Mazz (Yinhua); the mixture was decocted in a volume of 150 ml, cooled, bagged, and sealed to facilitate subsequent use.

### 2.2. Animal Experiments

#### 2.2.1. Animal Treatment

One hundred New Zealand White rabbits (female, 4-5 months old, 2.5–3.0 kg) were adaptively fed for one week. To establish a model of chronic inflammatory obstruction of the fallopian tube, a mixture of bacteria was formulated: *Escherichia coli*, *Staphylococcus aureus*, and *Streptococcus* were mixed at a ratio of 2 : 1 : 1 and diluted with saline to a concentration of 3 × 10^9^ CFU/mL. All strains were provided by the Central Laboratory of Comprehensive Practice Teaching Base of Yunnan University of Traditional Chinese Medicine. Sixty animals were selected randomly, and the bacterial mixture was injected into the uterus at the junction of the proximal tubal and the original segment, slowly injecting 0.05 ml bacterial suspension into bilateral fallopian tubes only once. Hysterosalpingography (HSG) was used to ensure a successful operation (HSG examination confirmed that the fallopian tube was blocked). After 15 days of modeling, the animals were divided into four groups: the model control (rabbit model, A), interventional therapy (B), medicine gavage (C), and enema treatment groups (D). The A and B groups were given normal feeding for two months. Each rabbit in the C group was at 10 mL/day gavage, and the D group was treated at 5 mL/day by enema for the same amount of time.

All animals were kept in a pathogen-free environment and fed ad libitum. The procedures for the care and use of animals were approved by the Ethics Committee of the Third People's Hospital of Yunnan, and all applicable institutional and governmental regulations concerning the ethical use of animals were followed. The approval number is No. 20200415.

#### 2.2.2. Determination of Biochemical Indexes

After two months of treatment, all animal samples were collected within one day. First, 10 mL of whole blood was gathered from the ear vein by negative-pressure blood collection, and serum was obtained by centrifugation after incubation at 4°C overnight and further used for determination of IL-1*β*, IL-6, IL-10, and TNF-*α* levels by ELISA kits.

#### 2.2.3. Transmission Electron Microscopy Observation

Fallopian tube lumen samples were collected from rabbits, fixed with glutaraldehyde, and then washed three times with PBS. After that, 1% osmic acid was used for fixation for 1 hour, and the samples were washed again with PBS. Anhydrous ethanol at concentrations of 50%, 70%, 80%, and 90% was used for gradient dehydration, and each concentration was used once for 10 min. The samples were returned to acetone for 10 minutes and soaked in the resin for 1 hour. Afterward, the specimens were soaked for 1 hour in a mixture of acetone and resin (1 : 1). Then, the samples were placed in resin overnight. The samples were picked out, placed in resin, heated to 45°C, and incubated for 48 hours. Finally, the samples were sectioned and stained with acetic acid oil and lead citrate for 10 minutes. All samples were observed by TEM.

#### 2.2.4. PCR Array and Quantitative Real-Time PCR Validation

For mRNA detection, the oviduct tissues were ground with liquid nitrogen and then disrupted with TRIzol to extract total RNA. Gene expression profiles were analyzed by a rabbit bone morphogenetic protein (BMP) qPCR array (Wcgene Biotech, Shanghai, China) according to the manufacturer's protocol. Data were analyzed using Wcgene Biotech software. Genes with fold changes greater than or less than 2.0 were considered to be of biological significance. To confirm the result of the PCR array, a StepOnePlus™ real-time PCR system (Thermo Fisher Scientific, the United States of America) was used to quantify the gene expression levels. The final qRT-PCR volume was 10 *μ*L, and the protocol was as follows: 95°C for 30 s and 40 cycles of 95°C for 5 s and 60°C for 30 s. Three independent samples were analyzed in triplicate.

### 2.3. Clinical Observation of the Treatment

#### 2.3.1. Patient Selection

The criteria for simple tubal obstruction infertility were as follows: (1) females of childbearing age who have a normal sex life, do not take contraceptive measures, and have not been pregnant for one year or more and whose spouse's reproductive function is normal; and (2) females of childbearing age whose serology and cervical secretions are normal, but who are still unable to get pregnant and have unilateral or bilateral tubal obstruction, hydrosalpinx, or tubal inflammation, as determined by hysterosalpingography (HSG).

The criteria for evaluating clinical efficacy were as follows: (1) the patient was pregnant within the past year, and HSG examination revealed that the affected fallopian tube was unobstructed and considered cured. (2) The affected fallopian tube was significantly improved after treatment, which means that the patients' condition was ameliorated. (3) If the fallopian tube was still blocked within half a year after treatment, the treatment was invalid.

From July 2010 to June 2016, a total of 163 patients diagnosed with oviduct obstruction infertility by HSG were selected. The patients were randomly divided into a hysteroscopy group and an intervention group, with 83 and 82 cases, respectively. All the above patients were treated in the Radiology Imaging Department of the third people's Hospital of Yunnan Province, No. 292, Beijing Road, Kunming, Yunnan Province, and were ethically approved.

#### 2.3.2. Procedure for the Intervention [20]

The operation was performed for 3–7 days after menstruation. The procedure was as follows: 30 mg ketorolac tromethamine and 10 mg raceanisodamine hydrochloride were injected intramuscularly half an hour before the operation, and 0.1% benzalkonium bromide was used for disinfection.

The position of the uterus was determined, the cervix was exposed and disinfected with iodine, and the probe was utilized to explore the depth of the uterine cavity. 10 to 15 ml of 76% compound meglumine diatrizoate was injected through a 12 F uterine catheter for HSG determination to confirm the shape of the uterine cavity and the location of the tubal obstruction.

A 5.5 F single-bend catheter was inserted after the catheter was withdrawn. After the 3 F catheter and 0.018 guidewires were combined, and the 5.5 F single-bend catheter entered the affected fallopian tube for dredging, the moving distance was approximately 2-3 cm, and the time was 1 min. Then, the guidewire was withdrawn, and compound meglumine diatrizoate was injected again. If it diffused into the pelvic cavity, it indicated that the recanalization was successful, and the images were collected.

During tubal recanalization, a mixture of 40,000 U gentamicin, 5 mg dexamethasone, 4000 U *α*-protease, and 10 ml normal saline was slowly injected through the catheter in 5 min. For the last 2 mL, the 3 F catheter was withdrawn, while the injection was pushed. The F catheter was withdrawn, and the contralateral side was dredged.

After 2 hours of observation, the patients could rest at home if they had no abdominal pain or vaginal bleeding. Antibiotics were routinely used within 3–5 days, and the patient's condition was closely observed.

#### 2.3.3. Combined Treatment with TCM

For one month after the operation, the patients were forbidden to have sex and take baths, and they were prescribed oral Chinese medicine and further retention enemas after the operation.

### 2.4. Data Analysis

The above data were collected and analyzed with SPSS 20.0. The chi-square test (*χ*^2^) was utilized to inspect and revise the statistics, whereas the measurement data were calculated as the mean (*X*) ± standard deviation (*s*). Moreover, a one-tailed *t* test was used, with the differences being significant only if the *P* value was <0.05.

## 3. Results

### 3.1. Observation by Transmission Electron Microscopy

Fallopian tubes from rabbits in the four groups were selected and observed with a transmission electron microscope (Figure 1). In the negative control group, The figure shows a typical a typical fallopian tube blockage in the negative control group, the number of cilia was significantly reduced, and the number of secretory granules was significantly increased (Figure 1(a)). In addition, the endoplasmic reticulum exhibited immense swelling, with shrinkage of the nuclear membrane and damage to the organelles (Figure 1(a)). After interventional recanalization treatment, despite the remarkable renewal of microvilli, there were still a large number of vacuoles, accompanied by shrinkage and dissolution of the nucleus and a decrease in the number of secretory cells (Figures 1(b) and 1(b)). Figures 1(c) and 1(d) show the condition of fallopian tube after different administration routes. Combining medicine gavage and interventional therapy, the length and diameter of ciliated cells increased, and the number was more than that of the above two groups. Secretory granules were also significantly reduced, and endoplasmic reticulum and nucleus showed no obvious damage (Figures 1(c) and 1(c)). However, compared with gavage, enema treatment has better therapeutic effect (Figures 1(d) and 1(d)).

### 3.2. Determination of Biochemical Indexes

As shown in Figure 2, the levels of IL-1*β*, IL-6, and TNF-*α*, three proinflammatory factors, were all reduced after the intervention. TCM combined with interventional therapy induced the strongest downregulation, especially in the enema treatment group, followed by gastric lavage with TCM and interventional therapy treatment alone (Figures 2(a)–2(c)). In contrast, the interventional therapies increased IL-10 expression in rabbits (Figure 2(d)), and enema with TCM was found to have the maximum effect. All the results indicated that, compared with fallopian tube intervention, recanalization combined with TCM could influence the secretion of cytokines and further affect the cure of tubal obstruction.

### 3.3. PCR Array

We collected oviduct tubes and examined the changes of genes in the TGF-*β* family to elucidate the expression level alterations that occur following an operation. Total RNA from oviduct tubes was isolated and evaluated by PCR array. The identities of 84 selected genes and the heatmap of the data for each sample are shown in Figure 3. The number of genes whose expression changed is summarized in Figure 4. The present study showed that the expression of 7 genes changed after treatment: BMP4, BMPR1A, SMAD4, KLF10, SMAD2, SMAD3, and SMAD7. More specifically, after combined treatment with the TCM preparation, the expression levels of BMP4, BMPR1A, SMAD4, KLF10, SMAD2, and SMAD3 were all increased, and SMAD7 showed the opposite pattern. These results suggest that TCM treatment can affect gene expression and further improve the condition of the fallopian tubes.

### 3.4. Analysis of the Tubal Patency Rate at 12 Months Postoperatively

As shown in Table 1, more than half of the patients in both groups had a postoperative unobstructed after the operation, and the tubal patency rate in the combined TCM enema group was substantially higher than the rate in the control group (81.9% vs. 53.1%), a difference that was statistically significant (*P*=0.015,  *P* < 0.05). However, at the same time, some patients' fallopian tubes are not completely unobstructed (34.9% vs. 18.3%, Interventional recanalization vs. combined medicine enema). Among them, the proportion of patients with partial fallopian tube obstruction was 22.9% vs. 13.4 (Interventional recanalization vs. Combined medicine enema), and the proportion of patients with complete obstruction was 22.9% vs. 13.4 (Interventional recanalization vs. Combined medicine enema). These data prove that traditional Chinese medicine combined with interventional recanalization can better improve the patency rate of fallopian tube.

## 4. Discussion

Tubal Obstructive Infertility is harmful to women's health, and inflammation is the main cause of tubal obstruction. Tubal obstruction is also accompanied by the changes of inflammatory factors. As the key proinflammatory cytokine, high expression of IL-6 can induce fibroblast proliferation, aggravate local pelvic adhesion and tubal injury, and eventually cause local tubal tissue adhesion, stenosis, and quince, leading to infertility [21, 22]. In addition, high expression of IL-1*β* can induce tissue injury and chronic inflammation, resulting in pelvic tissue adhesion and fibrosis [23–25]. Furthermore, TNF-*α* is closely related to tubal inflammatory injury and infertility [26, 27]. When tubal inflammation occurs, it induces the local immune system of the fallopian tube to secrete TNF-*α* continuously, promote an inflammatory reaction, aggravate damage to the fallopian tube and local pelvic adhesions, and stimulate the proliferation of fibroblasts, resulting in tubal narrowing and obstruction [9, 28, 29]. In this study, combination therapy significantly reduced the secretion of three proinflammatory factors, which shows that it can resist tubal inflammation and prevent tubal adhesion. In contrast, IL-10 is an important endogenous anti-inflammatory cytokine that is produced mainly by activated macrophages, and its effect may involve different feedback loops in the inflammatory response [8] and increase the levels of anti-inflammatory factors, which suggests that TCM may affect the secretion of inflammatory factors, reduce inflammatory reactions, alleviate tubal obstruction, and further promote the occurrence of pregnancy.

Oral administration of TCM is the most traditional method of administration. Many studies have asserted that oral TCM can produce an anti-inflammatory effect, which directly inhibits the release of a variety of inflammatory mediators and promotes the recovery of diseases [30–32]. However, it is often accompanied by the liver first-pass effect, which can reduce the bioavailability of the TCM. Compared with oral TCM administration, retention enema is an effective way to treat inflammation. Intestinal administration can cause the drug to be absorbed from the rectal mucosa directly to the lesion to inhibit the proliferation of connective tissue caused by salpingitis, resist the degeneration and necrosis of the mucosal epithelium, and inhibit inflammatory infiltration [31]. Yang Xinming et al. [33] proved that enema administration of Gexiazhuyu decoction has a better clinical effect than oral administration in the treatment of chronic pelvic inflammatory disease. Comparing the clinical effect of enema administration with that of oral administration for other TCMs also demonstrated identical results [34–36], which were equivalent to those of our study.

TGF-*β* is a receptor superfamily of polypeptide growth factors related to structure and function, including TGF-*β*, activin, bone morphogenetic proteins (BMPs), and growth differentiation factor (GDF). BMP4 is a member of BMPs, which is related to the transformation of primordial follicles to primary follicles [37]. There is a literature showing that the BMP4 ligand has a high affinity for the BMPR1A receptor [38]. Monsivais et al. [39] suggested that, as a type I receptor in the BMP/SMAD signaling pathway, the deletion of BMPR1A leads to infertility in mice. Additionally, BMPR1A can specifically bind to different types of ligands and plays an important role in the formation of the anterior pituitary, the development of ovarian granulosa cells, and the proliferation and differentiation of multifunctional stem cells during mammalian embryonic development [40–43]. After BMP4 binds to BMPR1A, it further activates the SMAD-dependent signaling pathway, which is a classical response to BMP. SMAD4 is a kind of comediator SMAD found in vertebrate, carries TGF-*β* signals into the nucleus, and plays an important role in mammalian ovarian follicle development, proliferation, and differentiation of granulosa cells, and reproductive performance, widely expressed in rat ovaries and mainly distributed in follicles [44–46]. In early development, SMAD4 is mainly expressed in primordial follicles and preantral follicles. With the maturation of the ovary, the expression of SMAD4 in stromal cells gradually increases [47]. In our study, combined therapy increased the expression of BMP4, further activated the BMP4/SMAD signaling pathway, promoted the development of primordial follicles, inhibited the apoptosis of oocytes, and improved the quality of oocytes.

Krüpple⁃like factor 10 (KLF10) is a rapidly expressed and activated early response gene that acts as a gene transcription repressor to inhibit SMAD7 gene expression and as a gene activator to induce SMAD2 gene expression. We found that KLF10 was upregulated after treatment and played a role in TGF-*β*-mediated cell growth control and differentiation. SMAD7 is a receptor inhibitory protein that has a negative feedback effect on the TGF-*β*/SMAD signal transduction pathway. Activated TGF-*β*1 phosphorylates receptor-activated SMADs, initiates the TGF-*β*/SMAD signal transduction pathway, and activates the inhibitory protein SMAD7. SMAD7 can inhibit the phosphorylation of SMAD2 and SMAD3 by TGF-*β*, increase the degradation of TGF-*β* R1 itself, and interrupt the signal transduction pathway [48, 49]. SMAD2 and SMAD3 are members of the SMAD protein family receptor regulation, and their main function is to participate in signal transduction in the TGF-*β* and activin signaling pathways. To date, research has revealed that SMAD2 and SMAD3 are involved in the upregulation of TGF-*β*1 expression and the production of PGE2, further participating in the occurrence and development of ovarian regulation of ovulation [50–52]. In addition, studies have shown that the fertility of SMAD2 and SMAD3 gene knockout mice is significantly reduced, and normal cumulus expansion and signal transduction between granulosa cells and oocytes cannot occur [53]. In general, TCM enema can affect the expression of genes in the TGF-*β*/SMAD signaling pathway. First, it significantly increases the expression level of KLF10, thereby downregulating the level of SMAD7 and further inducing the secretion of SMAD2/3, affecting normal follicular cell maturation and improving ovarian function.

A large number of researches have reported that TCM could alleviate or even cure female infertility, and there was little adverse reaction [54]. In order to confirm the effect of this TCM combined with interventional recanalization, we further proved it through clinical experiments. Due to the superiority of enema retention therapy in animal experiments, we compared it with interventional recanalization alone. The tubal patency rate in the postoperative 12 months in the combined therapy group (81.7%) was significantly higher than that of the interventional recanalization group (53.1%), which proves the conclusion obtained in animal experiments. In our study, we selected nine kinds of TCM composed prescription and used them on combination therapy. All these TCM have prominent anti-inflammatory and antibacterial effects [55–57], which may be the reason why this prescription is effective for tubal obstruction. Moreover, Danggui perceived enriches the blood, enhances blood circulation so as to alleviate pain, nourishes the liver, and regulates menstruation in Chinese Medicine [58]. Ezhu and Sanleng have also found the effect of promoting blood circulation and removing blood stasis, and they can be combined with moxibustion to treat chronic pelvic inflammatory disease [59]. In general, the therapeutic effect of this prescription on inflammatory tubal obstruction may be due to its excellent blood activating and anti-inflammatory effects. Thus, the theory of TCM combined with interventional recanalization in the treatment of tubal obstruction can be further promoted clinically. However, the goal of treatment is to make the patient pregnant; our study only focused on the patency of fallopian tube and did not pay further attention to the pregnancy rate. In addition, our study lacks certain clinical pharmacological evidence. Traditional Chinese medicine is composed of multiple drugs and contains a variety of chemical components, and its effects may not be limited to the anti-inflammatory and immune effects proved in this study. Therefore, we plan to further explore the clinical mechanism of this TCM preparation in future clinical studies.

## 5. Conclusion

In conclusion, TCM combined with interventional recanalization has a better effect on fallopian tube obstruction than interventional recanalization alone, which may be caused by the regulation of inflammatory factors and the inhibition of fallopian tube inflammation. Moreover, TCM can affect the TGF-*β*/SMAD and BMP/SMAD signaling pathways, promote the maturation of follicular cells, improve the ovarian environment, and thereby increase the pregnancy rate. It can also improve the patency rate of patients' fallopian tubes. These results also remind us that TCM can be used as a treatment for infertility caused by blocked fallopian tubes.

## Figures and Tables

**Figure 1:** Transmission electron microscopy of rabbit samples in four groups. (a) Negative control (rabbits untreated), (b) interventional therapy, (c) medicine gavage and interventional therapy group, and (d) enema treatment and interventional therapy group. Black Arrow: microvilli and cilia; White Arrow: secretory granules; Red Arrow: endoplasmic reticulum; Blue Arrow: nucleus. The magnification is shown in the figure.

**Figure 2:** Determination of IL-1*β*, IL-6, IL-10 and TNF-*α* levels in rabbit serum by ELISA. (a) IL-1*β*; (b) IL-6; (c) IL-10 and (d) TNF-*α*. (A) Negative control (rabbits untreated), (B) interventional therapy, (C) medicine gavage, and (D) enema treatment group. Moreover, the data are presented as the mean ± SD, and significant differences were represented as ^*∗*^*P* < 0.05,  ^*∗∗*^*P* < 0.01,  ^*∗∗∗*^*P* < 0.001 vs. the negative control group; *n* = 8.

**Figure 3:** Heat map showing the log (fold changes) in genes determined by PCR array analysis. Fold changes were calculated versus the solvent control average. The color scale ranges from red to blue, which denote up- and downregulated genes, respectively (for interpretation of the references to color in this figure legend, the reader is referred to the web version of this article). (A) Negative control (rabbits untreated), (B) interventional therapy, (C) medicine gavage, and (D) enema treatment group.

**Figure 4:** Expression levels of 7 different genes in rabbit oviduct tubes among groups. (A) Negative control (rabbits untreated), (B) interventional therapy, (C) medicine gavage, and (D) enema treatment group. The data are presented as the mean ± SD, and significant differences are represented as ^*∗*^*P* < 0.05,  ^*∗∗*^*P* < 0.01,  ^*∗∗∗*^*P* < 0.001.

**Table 1:** Analysis of the tubal patency rate (in nonpregnant patients) at 12 months postoperatively.

	Total of nonpregnant patients	Postoperative unobstructed	Postoperative partially obstructed	Postoperative obstructed	Patency rate (%)	95% CI
Interventional recanalization	83	44	19	10	53.1	(48.8, 71.8)
Combined medicine enema	82	67	11	4	81.7	(73.2, 90.3)

Patency rate = the number of postoperative unobstructed tubes/the number of follow-up patient tubes × 100%.

## Data Availability

All data generated or analyzed during this study are included in this published article.
